# Effects of microRNA-136 on melanoma cell proliferation, apoptosis, and epithelial–mesenchymal transition by targetting PMEL through the Wnt signaling pathway

**DOI:** 10.1042/BSR20170743

**Published:** 2017-09-07

**Authors:** Jiu-Jiang Wang, Zhi-Feng Li, Xiao-Jing Li, Zhao Han, Ling Zhang, Zhi-Jun Liu

**Affiliations:** Department of Dermatology, Affiliated Hospital of Hebei University of Engineering, Handan 056002, P.R. China

**Keywords:** Cell proliferation, Epithelial-mesenchymal transition, Melanoma cells, microRNA-136, PMEL, Wnt signaling pathway

## Abstract

The study aims to evaluate the effects of *miR-136* on the proliferation, apoptosis, and epithelial–mesenchymal transition (EMT) of melanoma cells by targetting premelanosome protein (PMEL) through the Wnt signaling pathway. After establishment of melanoma mouse models, melanoma (model group) and normal tissues (normal group) were collected. Immunohistochemistry was performed to determine PMEL protein concentration. Mouse melanoma cells were assigned into control, blank, negative control (NC), *miR-136* mimics, *miR-136* inhibitors, siRNA-PMEL, and *miR-136* inhibitors + siRNA-PMEL, LiC1 (Wnt signaling pathway activator), and siRNA-PMEL+ LiCl groups. MTT, Scratch test, Transwell assay, and flow cytometry were performed to measure cell proliferation, migration, invasion, and apoptosis. Quantitative real-time PCR (qRT-PCR) and Western blotting were performed to evaluate *miR-136*, PMEL, β-catenin, Wnt3a, Bcl-2, Bax, Caspase, E-cadherin, and N-cadherin expressions. PMEL is highly expressed in melanoma tissues. *MiR-136*, Bax, Caspase, and E-cadherin expressions decreased in the model group, whereas PMEL, β-catenin, Bcl-2, Wnt3a, and N-cadherin expressions increased. Bax, Caspase, and E-cadherin expressions increased in the *miR-136* mimics and siRNA-PMEL groups, whereas the expressions decreased in the *miR-136* inhibitors group and LiC1 group. PMEL, β-catenin, Bcl-2, Wnt3a, and N-cadherin expressions, cell proliferation, migration, and invasion decreased, and the apoptosis rate inceased in the *miR-136* mimics and siRNA-PMEL groups; whereas the tendencies were opposite to those in the *miR-136* inhibitors group and LiC1 group. In the siRNA-PMEL+ LiCl group, PMEL expression decreased. These findings indicated that overexpression of *miR-136* inhibits melanoma cell EMT, proliferation, migration, invasion, and promotes apoptosis by targetting PMEL through down-regulation of the Wnt signaling pathway.

## Introduction

Melanoma is a type of tumor cells that originates from melanocytes and it primarily develops in skin [1]. It has been reported that the main reasons for melanoma are genetic factors and UV radiation exposure [2]. In recent years, the incidence of melanoma has increased worldwide [3]. Approximately 200000 people are diagnosed with melanoma annually; melanoma causes approximately 80% deaths related to skin cancer [4,5]. Till date, although several therapeutic treatment options are available for melanoma such as chemotherapy, surgery, and immunotherapy, still the 5-year survival rate after operation is only 5–10% because of melanoma metastasis in those patients who underwent surgery [6,7]. Therefore, it is important to further investigate new preventive strategies and therapeutic methods to treat melanoma. In recent years, substantial studies revealed that miRNAs have an indispensable role in melanoma prognosis and metastasis [8].

MiRNAs refer to small non-coding RNA molecules, which induce gene silencing by degrading mRNAs or inhibiting translation by binding the 3′-UTR of its target gene [9]. Accumulated evidence revealed that miRNAs play vital roles in various biological processes, such as cellular proliferation, invasion, and apoptosis [10,11]. A study investigated that miRNAs and miRNA-target genes significantly influence human melanoma [12]. Premelanosome protein (PMEL), also known as PMEL17, silver, and gp100, is a kind of amyloidogenic protein, which is only expressed in pigment cells and causes the formation of physiological amyloid in melanosomes [13,14]. A recent study revealed that the critical PMEL domain had a significant impact on the formation of melanoma [15]. Wnt proteins constitute a family of secreted signaling molecules, regulating highly conserved pathways essential for development and drive oncogenesis in multiple human cancers when aberrantly activated [16]. In addition, it has been reported that the Wnt pathways serve as a potential target for treating cancers, because Wnts and downstream effectors play a crucial role in a variety of processes that are significant for cancer progression, such as metastasis, cell proliferation, and apoptosis [17–19]. Therefore, the present study was conducted to explore the modulatory effects of *miR-136* on the cell proliferation, epithelial–mesenchymal transition (EMT), and apoptosis of mouse melanoma cells by targetting PMEL through Wnt signaling pathway.

## Materials and methods

### Experimental animals

Forty male Kunming mice (aging 3-month-old and weighing 20 ± 2 g; specific-pathogen-free) were acquired from the Experimental Animal Center of Southern Medical University. All mice were acclimatized to laboratory conditions (1 week before the experiment): the humidity was 50–60% (22–24°C), the diurnal cycle was 12 h, with free access to food and water. All experimental procedures were strictly in accordance with the management and principles of use of the local experimental animals and abide by the *Declaration of Helsinki*.

### Selection of melanoma cell lines

The melanoma cell lines B16, A375, WM239, and WM451 were purchased from the Institute of Biochemistry and Cell Biology, Shanghai Institutes for Biological Sciences, Chinese Academy of Sciences (Shanghai, China). The cells were cultured in RPMI 1640 culture medium (SP1355, Shanghai Shifeng Biological Technology Co., Ltd., Shanghai, China) containing 10% FBS (Hyclone, Logan, Utah, U.S.A.), 100 U/ml of penicillin and 100 mg/ml streptomycin, and incubated at 37°C in a constant-temperature incubator (DHP-9162, Shanghai Jiecheng Lab Instruments Co., Ltd., Shanghai, China) along with 5% CO_2_. Fresh culture medium was replaced every 1 or 2 days. Once the cell confluence reached 80–90%, the cells were subcultured, and the third-generation cells were incorporated in further experimentation.

Quantitative real-time PCR (qRT-PCR) was performed to determine *miR-136* expression in the B16, A375, WM239, and WM451 cells. The total RNA was extracted with a TRIzol Extraction Kit (15596-018, Invitrogen, CA, U.S.A.). The ratio of *A*_260_/*A*_280_ and RNA concentration were measured by a Nanodrop Ultraviolet Spectrophotometer (2000, Thermo, Waltham, MA, U.S.A.), and the extracted RNA was preserved at –80°C. Reverse transcription was performed by First Strand cDNA Synthesis Kit (RR037A, Takara Biotechnology Inc., Dalian, China) to prepare the cDNA. The qRT-PCR RNA Test Kit was purchased from Applied Biosystems (NY, U.S.A.). The qRT-PCR experiment was conducted using an AM 1005 qRT-PCR system (AM1005, Invitrogen, CA, U.S.A.). Reaction conditions for *miR-136* were as follows: predenaturation at 95°C for 3 min, followed by 35 cycles denaturation at 95°C for 15 s, annealing at 60°C for 30 s,and extension at 72°C for 60 s. U6 was set as an internal reference for *miR-136* measurement. The relative expression of target gene [20] was measured by the 2^−ΔΔ*C*^_t_ method: ΔΔ*C*_t_ = *C*_t_ (target gene) (control group) – *C*_t_ (internal reference) (case group).

### Establishment of melanoma mouse models

Twenty mice were selected on random to establish melanoma mouse models (model group). The fur on left hind paw of the mouse was shaved off with a pair of ophthalmic scissors, followed by skin disinfection with 75% ethanol. B16 cells (1 × 10^5^) were extracted. The cell suspension (0.2 ml) was injected into the subcutaneous tissues of left hind paw. When the inoculated tumor cells became active tumor and its diameter reached close to 0.6 cm, the mice were killed and the tumor mass was separated. Another 20 mice were included in the normal group.

### Hematoxylin and Eosin staining

The melanoma tissues and normal tissues were fixed in 3% neutral formalin. The samples were embedded in paraffin, and prepared into tissue sections (5–8 μm). At first, the tissue sections were dewaxed by xylene twice, 5 min per time. Then, they were dehydrated with 100, 95, 80, and 75% ethanol for 1 min successively, and washed with water for 2 min. Then the sections were stained with Hematoxylin for 2 min, washed with water for 10 s, and separated by ethanol solution containing 1% hydrochloric acid for 10 s. After washing with distilled water for 1 min, the sections were stained with Eosin for 1 min. After washing with distilled water for 10 s, the sections were dehydrated with 95 and 100% ethanol twice, respectively, 1 min per time. Finally, after transparentizing with xylene, the sections were mounted in neutral balsam.

### Immunohistochemistry

The tissue samples were fixed with 10% formalin and embedded in paraffin. Serial sections (4 μm) were prepared, and were placed in an incubator at 60°C for 1 h. After drying, the sections were dewaxed by xylene three times, 10 min per time, and were then dehydrated by gradient alcohol of 95, 80, and 75% for 1 min, respectively. After washing with water for 1 min, the sections were incubated in 3% H_2_O_2_ (84885, Sigma, San Francisco, CA, U.S.A.) at 37°C for 30 min followed by another wash with PBS for 3 min, after which the sections were boiled in citrate buffer (0.01 M) at 95°C for 20 min. After the sections cooled down to room temperature, they were washed with PBS. The sections were blocked with normal sheep serum at 37°C for 10 min, and the primary antibody rabbit anti-mouse PMEL (dilution 1:500, ab137078, Abcam, Cambridge, MA, U.S.A.) was added. The sections were incubated at 4°C overnight, and washed with PBS. The secondary antibody goat anti-rabbit with horseradish peroxidase (DF7852, Shanghai Yaoyun Biotechnology Co., Ltd., Shanghai, China) was added to the samples followed by an incubation at room temperature for 30 min, then coloring with DAB (ab64238, Abcam, Cambridge, MA, U.S.A.). The samples were counterstained with Hematoxylin, and mounted. The primary antibody was replaced by PBS as the negative control (NC), and the normal mucous membrane was set as the positive control. Five high magnification (400×) views were selected on random in each slice. In each field, 100 cells were counted and the score was determined by the percentage of positive cells [21]. A cell was considered as positive (+) if the ratio between positive cells and total cells was over 10%, while the cell was considered negative (–) if the ratio between positive cells and total cells was less than or equal to 10%.

### Cell grouping and transfection

The cells were assigned into control (subcutaneous cells from normal mice), blank (transfected with no sequence), NC (transfected with *miR-136* NC), *miR-136* mimics (transfected with *miR-136* mimics), *miR-136* inhibitors (transfected with *miR-136* inhibitors), siRNA-PMEL (transfected with siRNA-PMEL), *miR-136* inhibitors + siRNA-PMEL (transfected with *miR-136* inhibitors and siRNA-PMEL), LiC1 (treated with Wnt signaling pathway activator) and siRNA-PMEL + LiCl groups.* MiR-136* mimic served as a type of endogenous miRNAs, which could enhance the expression function of the endogenous *miR-136* [22]. *MiR-136* inhibitor is a chemically modified inhibitor special to the specific target *miR-136* in cells [23]. Treated cells were seeded in a six-well plate 24 h before transfection. When the cell density grew to approximately 30–50%, the cells were transfected according to the instructions of Lipofectamine 2000 (11668-019, Invitrogen, CA, U.S.A.). Melanoma cells from the LiC1 group in the logarithmic growth phase were extracted and treated with 30 mmol/l LiCl for 1 day. In other groups, 250 μl serum-free Opti-MEM (51985042, Gibco, Gaitherburg, MD, U.S.A.) was applied to dilute 100 pmol blank, NC, *miR-136* mimics, *miR-136* inhibitors, *miR-136* inhibitors + siRNA-PMEL, and siRNA-PMEL (50 nM as the final concentration), and cells were mixed and incubated at room temperature for 5 min. The 250 μl serum-free Opti-MEM was applied to dilute 5 μl of Lipofectamine 2000 and cells were mixed and incubated at room temperature for 5 min. Both the aforementioned cells were mixed, incubated at room temperature for 20 min, and added into the well of a cell-culture plate. Cells were cultured at 37°C with 5% CO_2_ for 6–8 h, and then the medium was replaced. After culturing for 24–48 h, the cells were used for further experimentation.

### qRT-PCR

Total RNA of melanoma tissues and normal tissues was extracted with an miRNeasy Mini Kit (217004, Qiagen Company, Hilden, Germany). The primers of *miR-136*, PMEL, β-catenin, Wnt3a, Bcl-2, N-cadherin, Bax, Caspase, E-cadherin, and U6 were designed and synthesized by Takara Corporation (Takara Biotechnology Ltd., Dalian, China) (Table 1). Reverse transcription (10 μl) was conducted using PrimeScript RT Reagent Kit (RR036A, TaKaRa Biotechnology Ltd., Dalian, China) to prepare cDNA according to the instructions. The reaction conditions were as follows: reverse transcription was performed at 37°C three times, 15 min per time; the inactivation of reverse transcriptase was performed at 85°C for 5 s. The reaction liquid was extracted for conducting fluorescent quantitative PCR according to the instructions of the SYBR® Premix Ex Taq™ II Reagent Kit (RR820A, TaKaRa Biotechnology Ltd., Dalian, China). The reaction system included (50 μl): 25 μl SYBR® Premix Ex Taq™ II (2×), 2 μl forward primer, 2 μl reverse primer, 1 μl ROX Reference Dye (50×), 4 μl DNA template, and 16 μl ddH_2_O. ABI 7500 quantitative PCR system (7500, Applied Biosystems Inc., NY, U.S.A.) was used for qRT-PCR measurement. The reaction conditions were as follows: predenaturation at 95°C for 30 s, followed by 40 cycles of denaturation at 95°C for 5 s, annealing at 60°C for 30 s, and extension at 72°C for 30 s. U6 was set as the internal reference for the relative expression of *miR-136*, and GAPDH for the relative expressions of PMEL, β-catenin, Wnt3a, Bcl-2, N-cadherin, Bax, Caspase, and E-cadherin. The relative quantitation 2^−ΔΔ*C*^_t_ method was applied to calculate the relative transcription level of target genes (*miR-136, PMEL, β-catenin, Wnt3a, Bcl-2, N-cadherin, Bax, E-cadherin*, and *Caspase* mRNA): ΔΔ*C*_t_ = Δ*C*_t_ (case group) – Δ*C*_t_ (control group), Δ*C*_t_ = *C*_t_ (target gene) – *C*_t_ (internal reference) [20].

**Table 1:** qRT-PCR primer sequences

Genes	Sequences
*miR-136*	Forward: 5′-ACACTCCAGCTGGGACTCCATTTGTTTTG-3′
	Reverse: 5′-CTCAACTGGTGGTGTCGTGGAGTCGGCAAT-3′
*PMEL*	Forward: 5′-CCCCAGGAAACTGACGATGC-3′
	Reverse: 5′-AGCCACAGGAGGTGAGAGGAAT-3′
*β-catenin*	Forward: 5′-CTTGACAGGAAAGACAACGG-3′
	Reverse: 5′-GCTTCTACGGATCGAAACTG-3′
*Bcl-2*	Forward: 5′-ATCTTCTCCTTCCAGCCTGA-3′
	Reverse: 5′-TCAGTCATCCACAGGGCGAT-3′
*Wnt3a*	Forward: 5′-CCCAAGCTTTCCTTGGCTGTGGCACCC-3′
	Reverse: 5′-CCGCTCGAGCCTTGCAGGTGTGCACGTCA-3′
*Bax*	Forward: 5′-GAACAGATCATGAAGACAGGG-3′
	Reverse: 5′-CAGTTCATCTCCAATTCGCC-3′
*Caspase*	Forward: 5′-TGGTCTTGTGACTTGGAGGA-3′
	Reverse: 5′-TGGCTTCTTATTGGCACGAT-3′
*E-cadherin*	Forward: 5′-AGTTTACCCAGCCGGTCTTTGAG-3′
	Reverse: 5′-TCGGTGGCTGAGACCTTCATC-3′
*N-cadherin*	Forward: 5′-GGAATCCCGCCTATGAGTGG-3′
	Reverse: 5′-TTGGATCAATGTCATAATCAAGTGCTGTA-3′
*GAPDH*	Forward: 5′-TGACATCAAGAAGGTGGTGA-3′
	Reverse: 5′-TCATACCAGGAAATGAGCTT-3′
*U6*	Forward: 5′-CTCGCTTCGGCAGCACATATACT-3′
	Reverse: 5′-ACGCTTCACGAATTTGCGTGTC-3′

### Western blotting

Entire protein was obtained from the extracted tissues using RIPA Reagent Kit (R0010, Beijing Solarbio Science & Technology Co., Ltd., Beijing, China), and BCA method was used to measure the protein concentration. The proteins were separated by PAGE and then transferred on to nitrocellulose membranes, which were blocked with 5% BSA at room temperature for 1 h. The diluted primary antibody rabbit anti-mouse polyclonal antibodies PMEL (1:1000, ab137078), β-catenin (1:5000, ab32572), Bcl-2 (1:2000, ab32124), Wnt3a (1:3000, ab28472), Bax (1:2000, ab32503), Caspase (1:500, ab13847), E-cadherin (1:50, ab1416), N-cadherin (1:50000, ab18203) (Abcam, Cambridge, MA, U.S.A.) were added for overnight incubation at 4°C and washed with PBS for five times, 5 min per time. Goat anti-rabbit IgG antibody labeled by HRP (dilution 1:5000, Beijing Zhongshan Golden Bridge Biotechnology Co., Ltd., Beijing, China) was added; the membrane was immersed in ECL Luminous liquid (WBKLS0500, Pierce, Rockford, IL, U.S.A.) and observed completion by developing in a dark room and photography.

### Dual-luciferase reporter gene assay

The biological prediction website www.microRNA.org was used for the target gene analysis of *miR-163* and to verify if PMEL was the direct target gene of *miR-136*. The target sequence and mutant sequence were designed according to the sequence of *PMEL* mRNA in 3′-UTR binding to *miR-136*. After the chemosynthesis of the target sequence, restriction sites XhoI and NotI were added on each side, and cloned into PUC57 vector. Following the detection of positive clones and recombinant plasmids by DNA sequencing methods, the synthesized segment was subcloned into psiCHECK-2 vector, and was transfected by bacillus coli DH5α cells to intensify the vectors. The plasmids were extracted according to the instructions of the Omega Plasmid Mini Reagent Kit. The cells were seeded in a six-well plate with two plasmids, 10^5^/well. After cell attachment, the cells were transfected according to the aforementioned methods. After successful transfection, the cells were acquired and cultured for 48 h. The changes in luciferase activity of PMEL 3′-UTR, which were affected by *miR-136* were detected according to the method of the Dual-Luciferase Reporter Assay Reagent Kit provided by Genecopoeia (MD, U.S.A.). GloMax 20/20 Luminometer Luciferase Reporter Assay System (Promega, Madison, WI, U.S.A.) was used for testing the activity of dual luciferase. Each experiment was repeated thrice.

### MTT assay

After 48 h of cell transfection, cells were collected for cell count. The cells were seeded in a 96-well plate with a cell density of 3 × 10^3^ to 6 × 10^3^ cells in each well (0.1 ml; with six repeating wells). Experiments were conducted at 24, 48, and 72 h. The cells were cultured with MTT (5 mg/ml) at 37°C for 2 h. After extracting culture supernatant, 150 μl DMSO was introduced in each well. ELISA (NYW-96M, Beijing NYAW Instrument Co., Ltd., Beijing, China) was performed to test the absorbance value of each well. The optical density (OD) value of each hole at 570-nm site was measured. Each experiment was repeated thrice. The cell viability curve was drawn with the OD value set as the ordinate and the time point as the abscissa.

### Scratch test

Forty-eight hours after transfection, the cells were seeded in a six-well plate. DMEM serum-free medium was used after cell attachment. When the cell confluence reached close to 90–100%, spearhead (10 μl) was used to scratch the six-well plate perpendicular to its bottom, approximately 4–5 lines per well, to assure that the width of all the scratches was uniform. After washing with PBS three times, the scratched cells were removed and were cultured in an incubator. Scratch distance was determined under an inverted microscope at 0 and 24 h, and several fields were selected on random to take pictures. Three wells were set in each well and the experiment was repeated thrice.

### Transwell assay

Cells transfected for 48 h were digested in serum-free medium after starving for 24 h, and were washed with PBS twice. Then, the cells were then resuspended in serum-free medium Opti-MEMI (31985008, Nanjing SenBeiJia Biological Technology Co., Ltd., Jiangsu, China) containing BSA (10 g/l) to adjust the cell concentration to 3 × 10^4^ cells/ml. Transwell chambers were placed in a 24-well plate. The diluted Matrigel (40111ES08, Shanghai YASEN Biotechnology Co., Ltd., Shanghai, China) solution (1:8) was added in the upper chamber of basement membrane, and dried at room temperature. After digestion, the cells in the control, blank, NC, *miR-136* mimics, *miR-136* inhibitors, siRNA-PMEL, and *miR-136* inhibitors + siRNA-PMEL groups were washed with PBS twice. Cells were resuspended in RPMI 1640 medium, and cell density was adjusted to 1 × 10^5^ cells/ml. Cell suspension (200 μl) was added into the upper Transwell chamber coated with Matrigel, and RPMI 1640 medium (600 μl) with 20% FBS was introduced in the lower chamber. After culturing for 24 h, once the Transwell chamber was removed, cells on the internal surface of the lower chamber were wiped off with cotton buds. Cells were fixed in 4% paraformaldehyde for 15 min, followed by staining with 0.5 Crystal Violet solution (made up with methanol) for 15 min, and washing with PBS three times. Cells were photographed under an inverted microscope (XDS-800D, Shanghai Caikon Optical Instrument Co., Ltd., Shanghai, China) for five randomly selected views. The number of cells migrating through the Transwell chamber membrane was counted. Three wells were set in each group, and the experiment was repeated thrice to calculate the average value.

### Flow cytometry

After 48 h of transfection, the cells were collected, washed with PBS thrice, and centrifuged. The supernatant was discarded and the cells were resuspended in PBS after which they were readjusted to a concentration of approximately 1 × 10^5^/ml. The cells were fixed in 75% ethanol (–20°C precooled, 1 ml) at 4°C for 1 h, centrifuged for removing ice ethanol, washed with PBS twice, added with 100 μl RNase A, and kept away from light. The cells were allowed to rest in a water bath at 37°C for 30 min, and 400 μl PI (Sigma, SF, U.S.A.) was used for staining and mixing. After protecting the cells from direct light at 4°C for 30 min, flow cytometry was adopted to test the cell cycle by detecting red fluorescence at the excitation wavelength of 488 nm.

After 48 h of transfection, cells were digested by EDTA-free pancreatin and collected in flow tube. Cells were centrifuged to remove the supernatant. After washing with cooled PBS three times, the cells underwent centrifugation again to remove the supernatant. According to the instructions of the Annexin-V-FITC Cell Apoptosis Assay Kit (Sigma, SF, U.S.A.), Annexin-V-FITC/PI dye liquor was made with Annexin-V-FITC, PI, and HEPES (proportion; 1:2:50); and 1 × 10^6^ cells were resuspended in 100 μl dye liquor and evenly oscillated. After incubation at room temperature for 15 min, cells were added with HEPES buffer solution (1 ml), and evenly oscillated. Band pass filters of 525 and 620 nm, arisen by the excitation wavelength of 488 nm, were used to detect FITC and PI fluorescence, respectively for measuring cell apoptosis.

### Statistical analysis

All statistical analyses were conducted using SPSS 21.0 software (SPSS, Chicago, Illinois, U.S.A.). All measurement data were presented as mean ± S.D. One-way factor ANOVA was applied for comparison amongst multiple groups and *t* test was employed for comparing between two groups. *P*<0.05 was considered to be significantly different.

## Results

### Histopathological observations

The findings of Hematoxylin and Eosin (HE) staining (Figure 1) showed that compared with the control group, cells in the model group varied greatly in terms of size, with large volume and irregular shapes. Small amounts of melanin granules were observed in the cytoplasm of cells. Necrosis was observed in a large part of melanoma tissues, and a few inflammatory cells infiltrated melanoma mesenchyme and its peripheral tissues.

**Figure 1:** The results of Hematoxylin and Eosin staining (400×)

### Positive expressions of PMEL in melanoma tissues

Immunohistochemistry showed that PMEL protein in melanoma tissues was mainly distributed in the cytoplasm. The positive particles were brownish in color. The positive rate of PMEL protein in the normal group was (25.23 ± 2.48)%, while the positive rate of PMEL protein in the model group was (80.18 ± 6.24)%, which clearly indicated that the positive rate of PMEL protein in the normal group was much lower than that in the model group (*P*<0.05) (Figure 2).

**Figure 2:** The expression of PMEL protein in the normal group and model group (400×) (**A**) Expression of PMEL protein by immunohistochemistry; (**B**) positive rate of PMEL protein; *, *P*<0.05 compared with the normal group.

### The expressions of *miR-136*, Bax, Caspase, E-cadherin, PMEL, β-catenin, Bcl-2, Wnt3a, and N-cadherin in the normal group and model group

The results of qRT-PCR indicated that compared with the normal group, expressions of *miR-136*, Bax, Caspase, and E-cadherin significantly decreased in the model group, while the expressions of PMEL, β-catenin, Bcl-2, Wnt3a, and N-cadherin significantly increased (*P*<0.05).

The results of Western blotting showed that compared with the normal group, the expressions of Bax, Caspase, and E-cadherin significantly decreased in the model group, whereas the expressions of PMEL, β-catenin, Bcl-2, Wnt3a, and N-cadherin significantly increased (*P*<0.05) (Figure 3).

**Figure 3:** Expressions of Bax, Caspase, E-cadherin, PMEL, β-catenin, Bcl-2, Wnt3a, and N-cadherin in the normal group and model group (**A**) Histogram analysis of qRT-PCR; (**B**) histogram analysis of Western blotting; (**C**) protein banding pattern by Western blotting; *, *P*<0.05 compared with the normal group.

### *miR-136* specifically targetted PMEL

According to the online analysis software, there is a specific binding region between the PMEL gene sequence and *miR-136* sequence, therefore PMEL is one target gene of *miR-136* (Figure 4A). Luciferase assay was conducted to testify if PMEL was the target gene of miR-136 (Figure 4B). Compared with the NC group, the luciferase activity of wild-type Wt-*miR-136*/*PMEL* was inhibited in the *miR-136* mimics group (*P*<0.05), whereas the mutant 3′-UTR showed no significant changes (*P*>0.05). Therefore, it can be concluded that *miR-136* can specifically bind to the *PMEL* gene.

**Figure 4:** Verification of targetting relationship between* miR-136* and PMEL (**A**) The predicted binding site of *miR-136* on PMEL-3′-UTR; (**B**) luciferase activity determined by dual-luciferase reporter assay; *, *P*<0.05 compared with the NC group.

### The *miR-136* expression and mRNA expressions of Bax, Caspase, E-cadherin, PMEL, β-catenin, Bcl-2, Wnt3a, and N-cadherin in each group

The expression of *miR-136* in melanoma cell lines (B16, A375, WM239, and WM451) were evaluated by qRT-PCR. *MiR-136* was expressed in melanoma cell lines with different degrees, and the B16 cells with highest expression were chosen for further investigation (*P*<0.05) (Figure 5).

**Figure 5:** The *miR-136* expression and mRNA expressions of Bax, Caspase, E-cadherin, PMEL, β-catenin, Bcl-2, Wnt3a, and N-cadherin in each group (**A**) The differences in* miR-136* expression amongst the four cell lines; *, *P*<0.05 compared with B16; (**B,C**) the mRNA expressions in each group after transfection; *, *P*<0.05 compared with the control group; ^#^, both *P*<0.05, compared with the blank group and NC group.

In the model group, there was no obvious difference in the *miR-136* expression and mRNA expressions of Bax, Caspase, E-cadherin, PMEL, β-catenin, Bcl-2, Wnt3a, and N-cadherin between the blank group and NC group (*P*>0.05). In comparison with the blank and NC groups, the *miR-136* expression and mRNA expressions of Bax, Caspase, and E-cadherin in the *miR-136* mimics and siRNA-PMEL groups significantly increased (all *P*<0.05), whereas the mRNA expressions of PMEL, β-catenin, Bcl-2, Wnt3a, and N-cadherin significantly decreased (all *P*<0.05); *miR-136* expression increased markedly in the *miR-136* mimics group (*P*<0.05), whereas no significant difference was observed in the *miR-136* expression in the siRNA-PMEL group (*P*>0.05). The *miR-136* expression and mRNA expressions of Bax, Caspase, and E-cadherin significantly decreased in the *miR-136* inhibitors group (all *P*<0.05), while the mRNA expressions of PMEL, β-catenin, Bcl-2, Wnt3a, and N-cadherin significantly increased (all *P*<0.05). A significant reduction in the expression of *miR-136* was observed in the *miR-136* inhibitors + siRNA-PMEL group (*P*<0.05), whereas no significant change was observed in the mRNA expressions of Bax, Caspase, E-cadherin, PMEL, β-catenin, Bcl-2, Wnt3a, and N-cadherin (all *P*>0.05). The mRNA expressions of Bax, Caspase, and E-cadherin significantly decreased in the LiC1 group (all *P*<0.05), while the mRNA expressions of β-catenin, Bcl-2, Wnt3a, and N-cadherin significantly increased (all *P*<0.05) and there was no significant difference in *miR-136* expression and PMEL expression (*P*>0.05). In the siRNA-PMEL + LiC1 group, the PMEL expression decreased, while there were no significant changes in other indexes (all *P*>0.05) (Figure 5).

### The protein expressions of Bax, Caspase, E-cadherin, PMEL, β-catenin, Bcl-2, Wnt3a, and N-cadherin in each group after transfection

The findings of Western blotting (Figure 6) showed that compared with the control group, the protein expressions of Bax, Caspase, and E-cadherin in the other groups significantly decreased (all *P*<0.05), whereas the protein expressions of PMEL, β-catenin, Bcl-2, Wnt3a, and N-cadherin significantly increased (all *P*<0.05). No significant difference was observed between the blank group and NC group (*P*>0.05). In comparison with the blank and NC groups, the protein expressions of Bax, Caspase, and E-cadherin significantly increased in the *miR-136* mimics group and siRNA-PMEL group (all *P*<0.05), while the mRNA expressions of PMEL, β-catenin, Bcl-2, Wnt3a, and N-cadherin significantly decreased (all *P*<0.05). The protein expressions of Bax, Caspase, and E-cadherin significantly decreased in the *miR-136* inhibitors group (all *P*<0.05), while the protein expressions of PMEL, β-catenin, Bcl-2, Wnt3a, and N-cadherin significantly increased (all *P*<0.05). There were no significant changes in the protein expressions of Bax, Caspase, E-cadherin, PMEL, β-catenin, Bcl-2, Wnt3a, and N-cadherin in the *miR-136* inhibitors + siRNA- PMEL group (all *P*>0.05). The protein expressions of Bax, Caspase, and E-cadherin significantly decreased in the LiC1 group (all *P*<0.05), while the protein expressions of β-catenin, Bcl-2, Wnt3a, and N-cadherin significantly increased (all *P*<0.05) and there was no significant difference in PMEL expression (*P*>0.05). In the siRNA-PMEL + LiC1 group, the PMEL expression decreased, while there was no significant change in other indexes (all *P*>0.05).

**Figure 6:** The protein expressions of Bax, Caspase, E-cadherin, PMEL, β-catenin, Bcl-2, Wnt3a, and N-cadherin in each group after transfection (**A**) Protein expression in each group; (**B**) gray value analyzed by Western blotting; *, *P*<0.05 compared with the control group; ^#^, both *P*<0.05 compared with the blank group and NC group.

### *miR-136* inhibited cell proliferation of B16 cells

In comparison with the control group, the OD value increased at 48 and 72 h amongst the blank, NC, *miR-136* mimics, siRNA-PMEL, and *miR-136* inhibitors groups (all *P*<0.05). Compared with the blank group and NC group, the OD value increased in the *miR-136* inhibitors group and LiC1 group at 48 and 72 h after transfection, whereas it decreased in the *miR-136* mimics group and siRNA-PMEL group (all *P*<0.05). There was no significant change in OD value between the *miR-136* inhibitors + siRNA-PMEL group and siRNA-PMEL+ LiCl group (both *P>*0.05) (Figure 7).

**Figure 7:** Results of cell proliferation in each group at 24, 48, and 72 h after transfection *, *P*<0.05 compared with the control group, ^#^, *P*<0.05, compared with the blank group and NC group.

### *miR-136* inhibited cell migration of B16 cells

The results (Figure 8) showed that there was no evident difference in cell migration between the blank group and NC group (both *P*>0.05). In comparison with the control group, cell migration was stimulated in the model group (*P*<0.05). Compared with the blank group and NC group, cell migration was significantly inhibited in the *miR-136* mimics group and siRNA-PMEL group (both *P*<0.05), whereas it was stimulated in the *miR-136* inhibitors group and LiC1 group (both *P*<0.05). No significant change was observed in the *miR-136* inhibitors + siRNA-PMEL group and siRNA-PMEL + LiCl group (both *P*>0.05).

**Figure 8:** Effects of *miR-136* on cell migration of B16 cells in each group (**A**) Fusion of scratch gap in each group; (**B**) the number of migrant cells in each group; *, *P*<0.05 compared with the control group; ^#^, *P*<0.05, compared with the blank group and NC group.

### *miR-136* inhibited cell invasion of B16 cells

There was no evident difference in cell invasion between the blank group and NC group (both *P*>0.05). In comparison with the control group, cell invasion was stimulated in the model group (*P*<0.05). Compared with the blank group and NC group, cell invasion was significantly inhibited in the *miR-136* mimics group and siRNA-PMEL group (both *P*<0.05), while it was stimulated in the *miR-136* inhibitors group and LiC1 group (both *P*<0.05). No significant change was observed in the *miR-136* inhibitors + siRNA-PMEL group and siRNA-PMEL + LiCl group (both *P*>0.05) (Figure 9).

**Figure 9:** Effects of *miR-136* on cell invasion of B16 cells in each group (**A**) Cell invasion of each group under a microscope; (**B**) histogram of cell invasion; *, *P*<0.05 compared with the control group; ^#^, *P*<0.05 compared with the blank group and NC group.

### Cell cycle distribution after transfection

The cell percentage in the control, blank, NC, *miR-136* mimics, *miR-136* inhibitors, siRNA-PMEL, and *miR-136* inhibitors + siRNA-PMEL groups in G_0_/G_1_-phase was (88.70 ± 2.58)%, (70.81 ± 2.46)%, (71.79 ± 2.26)%, (80.78 ± 2.11)%, (61.52 ± 2.50)%, (79.62 ± 4.44)%, and (70.82 ± 1.33)%; and in S-phase was (1.33 ± 0.30)%, (20.95 ± 2.56)%, (22.58 ± 1.65)%, (12.96 ± 1.21)%, (31.37 ± 2.41)%, (12.82 ± 2.78)%, and (21.11 ± 1.94)%. In comparison with the control group, cell cycle distribution reduced (cell percentage decreased) in G_0_/G_1_-phase in the blank, NC, *miR-136* mimics, *miR-136* inhibitors, siRNA-PMEL, and *miR-136* inhibitors + siRNA-PMEL groups, while the cell cycle distribution increased (cell percentage increased) in S-period (all *P*<0.05). Compared with the blank group and NC group, cell cycle distribution was significantly increased (cell percentage increased) in G_0_/G_1_-phase, whereas it significantly decreased (cell percentage decreased) in S-phase in the *miR-136* mimics group and siRNA-PMEL group (all *P*<0.05), while it evidently decreased (cell percentage decreased) in G_0_/G_1_-phase, but it significantly increased (cell percentage increased) in S-phase in the *miR-136* inhibitors group and LiC1 group (both *P*<0.05). No evident change was observed in the *miR-136* inhibitors + siRNA-PMEL group and siRNA-PMEL + LiCl group (both *P*>0.05). No marked difference was observed in G_2_-phase in each group (*P*>0.05) (Figure 10).

**Figure 10:** Effects of *miR-136* on cell cycle distribution of B16 cells in each group (**A**) Cell cycle distribution in each group; (**B**) rate of cell cycle distribution in each group; *, *P*<0.05, compared with the control group;^ #^, *P*<0.05, compared with the blank group and NC group.

### *miR-136* promoted cell apoptosis of B16 cells

In comparison with the control group, the apoptosis rate significantly and successively decreased in the blank, NC, *miR-136* mimics, *miR-136* inhibitors, siRNA-PMEL, and *miR-136* inhibitors + siRNA-PMEL groups (all *P*<0.05). Compared with the NC and blank groups, apoptosis rate significantly increased in the *miR-136* mimics group and LiCi group (both *P*<0.05), while it evidently decreased in the *miR-136* mimics group and siRNA-PMEL + LiC1 group (both *P*<0.05). No significant difference was observed in apoptosis rate between the *miR-136* inhibitors + siRNA-PMEL, blank, and NC groups (all *P*>0.05) (Figure 11).

**Figure 11:** Effects of *miR-136* on cell apoptosis rate of B16 cells in each group (**A**) Cell apoptosis chart in each group; (**B**) apoptosis rate in each group; *, *P*<0.05 compared with control group; ^#^, *P*<0.05 compared with the blank and NC groups.

## Discussion

EMT is a common life-threatening melanoma, characterized by poor prognosis for patients [5]. It has been reported that deregulation of miRNAs is involved in a variety of human diseases, including cancer [24]. To elucidate the mechanism of miR-136 in melanoma, the present study was performed to examine the modulatory effects of *miR-136* by targetting PMEL via down-regulation of Wnt signaling pathway in mouse melanoma cells. Collectively, the study came to a conclusion that *miR-136* could attenuate cell proliferation and EMT, and stimulate apoptosis of mouse melanoma cells by targetting PMEL via down-regulation of Wnt signaling pathway.

The present study showed that decreased *miR-136* in mouse melanoma cells, was linked to the occurrence and development of melanoma. A previous study investigated that there are approximately half the number of miRNAs located in the chromosomal areas, which are amplified or deleted frequently in human cancer cells [25]. MiRNAs, relying on their downstream targets, are able to inhibit oncogenes [26]. Some miRNA family members have been proven to inhibit melanoma cell proliferation and invasion by regulating their target genes [27,28]. Our current data revealed that up-expressed miR-136 inhibited melanoma cell proliferation, migration, and invasion, and stimulated apoptosis. Moreover, accumulated evidence showed that *miR-136* served as a suppressor in the occurrence and development of various human cancers, and it may provide a therapeutic method in predicting and treating human cancers [29,30]. For instance, Haapa-Paananen et al. [31] investigated that *miR-136* reduced in human glioma cells and stimulated cell apoptosis of glioma cells via inhibition of AEG-1 and Bcl-2 [32]. A previous study showed that *miR-136* had a tumor-suppressive impact on breast cancer cells by targetting PTEN, a tumor inhibitor [33].

Our findings signified that PMEL expression was much higher in melanoma tissues compared with normal tissues, and *miR-136* suppressed mRNA and protein expressions of PMEL. PMEL is a type of transmembrane glycoprotein, which plays an important role in normal melanosome biogenesis pathway [34]. The present study also indicated that in the siRNA-PMEL group melanoma cell proliferation, migration, and invasion significantly reduced, while the rate of apoptosis increased. It is known that PMEL has a crucial role in the maturation of melanosome, which emphasizes on the different levels of hypopigmentation of PMEL mutations in animal models [35]. A previous study showed that the genetic mutations directly effected melanosomal function, which consequently not only effected pigment cell migration, differentiation, and survival, but also impacted the interference of biogenesis of melanoma, transfer to keratinocytes, and then into color variations of skin, eyes, or hair [36]. It has been previously investigated that melanosome elongation is vital for PMEL-dependent fibril formation during biogenesis of mammalian melanosome in melanocytes, which showed that PMEL had a crucial impact on melanoma formation [37,38]. Therefore, the present study reveals that targetting PMEL may provide a promising method for treating melanoma.

Our study also showed that *miR-136* inhibited the mRNA and protein expressions of β-catenin, Bcl-2, Wnt3a, and N-cadherin. The Wnt signaling pathway comprises a large number of ligands, which are signaling molecules in cell’s fate determination and can be assigned to receptors, co-receptors, and regulatory components [39–41]. The Wnt pathway has an effect on various cellular processes, such as proliferation, differentiation, apoptosis, and cell motility [42]. Tissue homeostasis, growth, and differentiation are indispensable for the Wnt signaling pathway [43]. Otherwise, aberrant Wnt signaling can lead to the abnormal development of a disease, and significantly influence the occurrence and progression of human cancers [17,44]. The first relation observed between the Wnt pathway and human cancer was due to initial recognition of mouse mammary oncogene *int-1*, which is regarded as a homolog of the *Drosophila* wingless (*Wg*) gene, bringing about the portmanteau family designation of ‘Wnt’ [45]. Constitutive activation of Wnt pathway, due to mutations of essential Wnt pathway genes, was considered as a feature of various human cancers including melanomas [46]. Moreover, some preceding studies investigated that activation of Wnt/β-catenin pathway greatly effected the inhibition of melanoma cell proliferation and stimulated apoptosis [47,48].

In addition, the current study also revealed that increased *miR-136* expression suppressed N-cadherin, but promoted mRNA and protein expressions of E-cadherin, which were outstanding hallmarks of EMT [49]. EMT development is affected by various factors such as interplay of miRNAs and aberrant activity of the Wnt/β-catenin pathway [50]. For instance, up-regulated *miR-200a* could suppress tumor cell growth, invasion, and EMT through increasing the expression of E-cadherin and reducing the expression of N-cadherin and β-catenin [51]. To conclude, *miR-136* decreased in melanoma, while PMEL was highly active in melanoma and consequently affected the development and progression of melanoma by regulating Wnt expression. Thus, the identification of *miR-136* down-regulating PMEL and the Wnt signaling pathway in melanoma may assist in unveiling and understanding the potential molecular mechanisms of melanoma and may aid in providing new prognostic markers for treating melanoma in the future. For complete understanding of the specific mechanisms of *miR-136* targetting PMEL via Wnt signaling pathway, further studies are required.

## Abbreviations

DMEM: Dulbecco's modified Eagle medium
EMT: epithelial–mesenchymal transition
NC: negative control
OD: optical density
PMEL: premelanosome protein
qRT-PCR: quantitative real-time PCR
